The article "Prenatal Prediction of Fetal Growth Restriction and Postnatal Outcomes by Ultrasound Assessment of Fetal Myocardial Performance Index and Blood Flow Spectrum" was retracted in 2023. Reasons: suspected computer-generated content; unreliable results or conclusions; concerns about the data; concerns about the results or conclusions.

# Prenatal Prediction of Fetal Growth Restriction and Postnatal Outcomes by Ultrasound Assessment of Fetal Myocardial Performance Index and Blood Flow Spectrum

**DOI:** 10.1155/2022/4234137

**Published:** 2022-05-05

**Authors:** Yanchun Ma, Chunmin Li, Yan Wang, Hong Zhang

**Affiliations:** ^1^Comprehensive Examination Department, Children's Hospital of Shanxi, Taiyuan, China; ^2^Health Services and Management, Shanxi University of Chinese Medicine, Jinzhong, China

## Abstract

**Objective:**

Fetal growth restriction (FGR) affects 5% to 10% of newborns and is a major determinant of perinatal morbidity and mortality. Myocardial performance index (MPI), also known as the Tei index, is a useful, noninvasive, and Doppler-derived myocardial performance tool for fetal cardiac function evaluation. The purpose of the study is to evaluate ultrasonic prediction on FGR and postnatal outcomes using MPI and blood flow spectrum.

**Methods:**

This retrospective study included 240 pregnant women developing FGR and 240 healthy pregnant women. The blood flow spectrum of middle cerebral artery (MCA), umbilical artery (UA), and ductus venous including systolic to diastolic ratio (S/D), resistant index (RI), pulse index (PI), and peak ventricular systolic velocity/atrial contraction valley velocity (S/a) were examined using the GE Voluson E8 ultrasound system.

**Results:**

The MPI, S/D, RI, PI of UA, and S/a were all higher but S/D, RI, and PI of MCA were lower in the FGR group than those in the control group (*P* < 0.001). The MPI, S/D, RI, PI of UA, S/D, RI, PI of MCA, and ductus venous S/a yielded AUC of 0.813, 0.835, 0.791, 0.804, 0.789, 0.796, 0.803, and 0.784 when they were used to predict the incidence of FGR. Of note, the pregnant women with poor pregnancy outcomes exhibited higher values of MPI, S/D, RI, PI of UA, and S/a with lower scores of 1 min Apgar concomitant with lower values regarding S/D, RI, and PI of MCA than those with favorable pregnancy outcomes (*P* < 0.001). The MPI (*r* = −0.623), S/D (*r* = −0.660), RI (*r* = −0.601), PI (*r* = −630) of UA, and S/a (*r* = −0.573) shared negative correlations with 1 min Apgar scores (*P* < 0.001). Of note, the S/D (*r* = 0.562), RI (*r* = 0.597), and PI (*r* = 0.619) of MCA were positively correlated with 1 min Apgar scores (*P* < 0.001). It was revealed that the MPI, S/D, RI, PI of UA, S/D, RI, PI of MCA, and ductus venous S/a yielded AUC of 0.806, 0.833, 0.774, 0.788, 0.807, 0.729, 0.748, and 0.770 when they were used to predict the incidence of poor pregnancy outcomes for pregnant women developing FGR.

**Conclusion:**

Our study demonstrates good ultrasonic prediction on FGR and postnatal outcomes using MPI and blood flow spectrum.

The article "Prenatal Prediction of Fetal Growth Restriction and Postnatal Outcomes by Ultrasound Assessment of Fetal Myocardial Performance Index and Blood Flow Spectrum" was retracted in 2023. Reasons: suspected computer-generated content; unreliable results or conclusions; concerns about the data; concerns about the results or conclusions.

## 1. Introduction

Fetal growth restriction (FGR), also known as intrauterine growth restriction, refers to the fetal fails to reach its intrauterine growth and development potential due to impaired placental function. FGR is a common pregnancy complication which contributed to various adverse perinatal outcomes [1], such as premature birth and intrapartum asphyxia, as well as health defects in adulthood, including impaired neurological and cognitive development and cardiovascular or endocrine diseases. FGR is associated with higher risk of perinatal mortality, accounting for 30% of stillborn infants [2]. Although the use of its definition affected the prevalence of FGR, FGR has been reported to be occurred in 5–10% of pregnancies [3]. Attempts have been made in elaborating definition of FGR, such as ultrasonography estimated fetal weight below the 10th percentile of gestational age, which was proposed by American College of Obstetrics and Gynecology and is commonly used [4]. FGR is frequently associated with placental insufficiency, and for those whose weight is lower than the 10th percentile of gestational age based on their genetic growth potential, they are appropriately described as a fetus smaller than gestational age instead of FGR [5].

The earliest uterine artery Doppler study revealed that the prediction rate of FGR was 15.4%, and the prediction rate of early-onset FGR was higher, with a sensitivity of 39.2% [6]. Prospective measurement of uterine height might be helpful in FGR screening. However, the sensitivity of this method can be affected by various factors such as body mass index, parity, maternal bladder volume, and amniotic fluid index [7, 8]. The pathological mechanism of FGR is complex and placental dysfunction is the main factor leading to FGR. Numerous studies have shown that fetal hemodynamic abnormalities are the main pathological reasons, which mostly occur in the umbilical artery (UA), middle cerebral artery (MCA), and venous ductus [9, 10]. Under normal circumstances, placental vascular resistance gradually decreases during pregnancy, and this trend will be reversed when placental dysfunction occurs. UA Doppler reflects placental vascular resistance [11].

In recent years, the Doppler technology has developed and popularized rapidly. It can intuitively show the direction of blood flow and effectively reflect the changes of fetal hemodynamics by measuring relevant parameters. Now, it has become an important means to monitor fetal blood circulation. Fetal hemodynamics abnormalities affect the fetal heart function to a certain extent [12]. The myocardial performance index (MPI), also known as the Tei index, was proposed by Tei in 1995, and modified MPI was a reliable index to assess fetal heart function under variety of pregnancy conditions including FGR [13, 14]. However, there are not many clinical reports on the predictive value of MPI on FGR pregnancy outcome. Based on this, this study evaluated MPI, blood flow spectrum of MCA, UA and ductus venosus by ultrasound, in order to provide objective data support for clinical prediction of FGR and adverse pregnancy outcomes.

The article "Prenatal Prediction of Fetal Growth Restriction and Postnatal Outcomes by Ultrasound Assessment of Fetal Myocardial Performance Index and Blood Flow Spectrum" was retracted in 2023. Reasons: suspected computer-generated content; unreliable results or conclusions; concerns about the data; concerns about the results or conclusions.

## 2. Methods

### 2.1. Study Subjects

This retrospective study included 240 pregnant women developing FGR and 240 healthy pregnant women who were given examinations at our hospital between January 2019 and December 2021 and approved by the Institutional Review Board of our hospital. Each pregnant woman signed an informed consent form before study enrollment. The diagnostic of FGR was confirmed by at least two examinations [15]: (i) an estimated fetal weight (EFW) at or below the 3^rd^ percentile compared to normal fetal weight for gestational age, or as fetuses with of an EFW at or below the 10th percentile; (ii) an abnormal Doppler or having a growth restriction in subsequent scans crossing centiles by more than two quartiles. Healthy pregnant women must have normal fetal weight and abdominal circumference for gestational age, without hyperemesis gravidarum or gestational hypertension, and the fetus must develop well with normal placenta and amniotic fluid volume, no evidence of structural malformations on the Doppler ultrasound. All included pregnant women had singleton pregnancy, with maternal age 18 years or over. Exclusion criteria were as follows: (i) chromosomal abnormalities, known aneuploidy, fetal cardiac anomaly, major/multiple congenital anomaly suggesting a syndromal cause for FGR; (ii) history of drug administration at early pregnancy or history of high-dose of radiation; (iii) abnormal umbilical cord insertion or single umbilical artery; (iv) fetal arrhythmia; (v) severe cognitive impairments or mental illness; (vi) unavailability of perinatal outcome data.

### 2.2. Conventional Ultrasonic Examination

All pregnant women were examined in the supine position by one of two sonographers with a GE Voluson E8 ultrasound system (GE Healthcare, Zipf, Austria) equipped with a transabdominal curvilinear transducer of frequency 2–5 MHz. The biparietal diameter (BPD), head circumference (HC), abdominal circumference (AC), and femur and humerus length (FL and HL) of the fetus were measured. The presence of structural malformations, placental development, and amniotic fluid volume was recorded. Gestational age was calculated according to last menstrual period and confirmed by first-trimester ultrasound examination.

The article "Prenatal Prediction of Fetal Growth Restriction and Postnatal Outcomes by Ultrasound Assessment of Fetal Myocardial Performance Index and Blood Flow Spectrum" was retracted in 2023. Reasons: suspected computer-generated content; unreliable results or conclusions; concerns about the data; concerns about the results or conclusions.

The pregnant women held their breath and the fetus was in quiescent condition. The MPI was performed on a cross-sectional plane of fetal thorax at the level of four chambers view with an apical projection. The angle of insonation was adjusted to less than 30°. The Doppler velocity was set at 15 cm/s, with WMF of 90 Hz and lowest gain color and mechanical and thermal indices less than 1. A Doppler sample volume size of 3 mm was placed at the internal leaflet of the mitral valve or tricuspid valve, with the pulsed Doppler trace including the positive waveform (E and A waveform) and the negative waveform (aorta or pulmonary artery waveform). The isovolumic contraction time (ICT) was determined from the beginning of the mitral valve closure to the aortic valve opening, IRT was measured from the aortic valve closure to the mitral valve opening, and ejection time (ET) was measured at the period from the aortic valve opening to closure. The MPI was estimated from (ICT + IRT)/ET.

The blood flow spectrum of middle cerebral artery (MCA) and umbilical artery (UA), including systolic to diastolic ratio (S/D), resistant index (RI), and pulse index (PI) was examined using GE Voluson E8 ultrasound system. The ductus venous blood flow examination was performed on the median sagittal plane or oblique section near the upper abdomen of the fetus. The long axis of umbilical vein was clearly displayed and the transducer was traced to the fetal head. Once the brightness of ductus venous is significantly greater than the color blood flow signal of peripheral vein on the color Doppler, sampling began at the ductus venous. The sound beam was maintained basically parallel to the direction of blood flow, and the angle of insonation was adjusted to less than 30°. The peak ventricular systolic velocity/atrial contraction valley velocity (S/a) was measured. The pregnant women held their breath and the fetus was in quiescent condition. Each parameter was tested in triplicates to obtain the average.

### 2.3. Statistical Analysis

The measurement data were analyzed for their homogeneity of variance and normal distribution using Bartlett's and Kolmogorov–Smirnov's test, respectively, and then reported as the mean ± standard deviation. Two-groups comparison of measurement data was performed by independent sample *t*-test. Frequencies and percentages were reported for categorical values. Pearson correlation coefficients were used to test MPI, S/D, RI, PI of MCA and UA, S/a, and 1 min Apgar scores. The area under the receiver operating characteristic (ROC) curve (AUC) was used as a performance measure of MPI, S/D, RI, PI of MCA and UA, S/a in predicting the occurrence of FGR. SPSS 22.0 software (IBM, USA) was employed for data analysis. A *P*-value less than 0.05 indicates statistically significant difference.

The article "Prenatal Prediction of Fetal Growth Restriction and Postnatal Outcomes by Ultrasound Assessment of Fetal Myocardial Performance Index and Blood Flow Spectrum" was retracted in 2023. Reasons: suspected computer-generated content; unreliable results or conclusions; concerns about the data; concerns about the results or conclusions.

## 3. Results

### 3.1. Demographics of Study Subjects

This retrospective study consisted of FGR group (242 pregnant women developing FGR) and control group (242 healthy pregnant women). The pregnant women in the FGR group aged from 23 to 39 years, with a mean age of (30.02 ± 3.25) years. The gestational age in the FGR group ranged from 32 to 36 weeks (34.28 ± 0.58) and the pregnancy times ranged from 0 to 2 times (1.44 ± 0.23). The pregnant women in the control group aged from 22 to 40 years, with a mean age of (30.10 ± 2.92) years. The gestational age in the control group ranged from 32 to 36 weeks (34.32 ± 0.60) and the pregnancy times ranged from 0 to 3 times (1.46 ± 0.26). The two groups were comparable due to no significant difference in maternal age, gestational age, and pregnancy times (*P* > 0.05).

### 3.2. Predictive Performance of MPI and Blood Flow Spectrum in FGR

As shown in Table 1, the MPI, S/D, RI, PI of UA, and S/a were all higher in the FGR group than those in the control group (*P* < 0.001). The FGR group showed lower values regarding S/D, RI, and PI of MCA than the control group (*P* < 0.001). When the MPI, S/D, RI, PI of UA and MCA, and S/a were used to predict the incidence of FGR, the AUCs with 95%CI and cutoff values were obtained and are listed in Table 2. The ROCs of MPI, S/D, RI, PI of UA and MCA, and S/a used to predict the incidence of FGR are depicted in Figure 1. Results showed that the MPI, S/D, RI, PI of UA, S/D, RI, PI of MCA and ductus venous S/a yielded AUC of 0.813, 0.835, 0.791, 0.804, 0.789, 0.796, 0.803, and 0.784 when they were used to predict the incidence of FGR.

### 3.3. Association between the MPI, Blood Flow Spectrum, and Pregnancy Outcomes

There were 33 pregnant women with poor pregnancy outcomes in the FGR group, including 10 cases of fetal death intrauterus, 16 cases of respiratory distress syndrome, 5 cases of metabolic acidosis, and 2 infants died during the neonatal days. Univariate analysis according to pregnancy outcomes, it was found that the MPI, S/D, RI, PI of UA, and S/a were all higher in pregnant women with poor pregnancy outcomes than those with favorable pregnancy outcomes (*P* < 0.001, Table 3). Of note, the pregnant women with poor pregnancy outcomes exhibited lower scores of 1 min Apgar concomitant with lower values regarding S/D, RI, and PI of MCA than those with favorable pregnancy outcomes (*P* < 0.001).

### 3.4. MPI and Blood Flow Spectrum Were Correlated with 1 min Apgar Scores

Pearson correlation coefficients were used to evaluate correlations between MPI, S/D, RI, PI of MCA and UA, S/a, and 1 min Apgar scores. The MPI (*r* = −0.623), S/D (*r* = −0.660), RI (*r* = −0.601), PI (*r* = −630) of UA, and S/a (*r* = −0.573) shared negative correlations with 1 min Apgar scores (*P* < 0.001). Of note, the S/D (*r* = 0.562), RI (*r* = 0.597), and PI (*r* = 0.619) of MCA were positively correlated with 1 min Apgar scores (*P* < 0.001).

The article "Prenatal Prediction of Fetal Growth Restriction and Postnatal Outcomes by Ultrasound Assessment of Fetal Myocardial Performance Index and Blood Flow Spectrum" was retracted in 2023. Reasons: suspected computer-generated content; unreliable results or conclusions; concerns about the data; concerns about the results or conclusions.

### 3.5. Predictive Performance of MPI and Blood Flow Spectrum in Pregnancy Outcomes

When the MPI, S/D, RI, PI of UA and MCA, and S/a were used to predict the incidence of poor pregnancy outcomes for pregnant women developing FGR, the AUCs, and cutoff values were obtained and are listed in Table 4. The ROCs of MPI, S/D, RI, PI of UA and MCA, and S/a used to predict the incidence of poor pregnancy outcomes for pregnant women developing FGR are depicted in Figure 2. It was revealed that the MPI, S/D, RI, PI of UA, S/D, RI, PI of MCA and ductus venous S/a yielded AUC of 0.806, 0.833, 0.774, 0.788, 0.807, 0.729, 0.748, and 0.770 when they were used to predict the incidence of poor pregnancy outcomes for pregnant women developing FGR.

## 4. Discussion

The prevalence of FGR was one of the reasons leading to increased poor pregnancy outcomes. It was the second leading cause of perinatal death of fetus, which was strongly associated with placental dysfunction [16]. Therefore, effective screening in FGR and early interventions are of great significance to improve pregnancy outcome.

As a result of presenting features of no damage, the noninvasive, high-resolution, ultrasonography method describes better main anatomical structure of fetus and is widely used in obstetric examination [17, 18]. Fetal umbilical artery and middle cerebral artery are the first affected vessels when FGR occurs [19]. Umbilical artery is an important link between maternal blood system and fetal blood system. Its hemodynamic changes are related to pathological changes of placenta. The umbilical artery resistance gradually decreases and the blood flow increases as a result of development and maturity of the placenta. The process is conducive to ensuring the demands of the fetus for normal growth and development [20]. The study presented by Aditya et al. has manifested that S/D that is more than 3.00 indicates fetal hypoxia [21]. It was reported that the PI of UA decreased with the increase of gestational age in normal pregnancies, and abnormally low PI of UA might be associated with adverse pregnancy outcomes [22]. Ciobanu et al. demonstrated that the median PI of UA decreased linearly with gestational age from 20 to 42 weeks [23]. The middle cerebral artery is the source of blood supply to the brain, and its blood flow changes objectively show the state of fetal cerebral blood circulation. It was reported that in the normal fetal situation, the average S/D ratio was 3.5 in the 40th week, and RI value decreased to 0.67 in the third trimester [24]. In our study, we compared S/D, RI, PI of UA and MCA. It was observed that compared with the control group, these values of UA were higher and these values of MCA were lower in the FGR group. This study confirmed that S/D, RI, PI of UA, and S/D, RI, PI of MCA yielded AUC of 0.835, 0.791, 0.804, 0.789, 0.796, 0.803, respectively when these values were used to predict the incidence of FGR. It is suggested that the monitoring of blood flow spectrum of UA and MCA by ultrasound is expected to be an important methods to predict FGR. The results we found might be induced by the changes of maternal placental blood flow resistance. The blood flow resistance of UA increases with the increase of blood flow resistance placenta in FGR, leading to the rise of PI, RI and S/D of UA and the decline of blood oxygen entering the placenta, followed by aggravation of intrauterine hypoxia and decrease of PI, RI and S/D of MCA. This study also determined the MPI between the two groups. The results indicated that the FGR group had higher value of MPI than the control group and MPI yielded AUC of 0.813 in predicting the incidence of FGR. These findings were supported by another research revealing late-onset FGR group showed increased MPI compared with the control fetuses, and increased MPI contributed to adverse outcomes [14]. Furthermore, early-onset and late-onset FGR groups both showed elevated modified MPI. The sensitivity and specificity of MPI for prediction of bad consequences in these two groups were 60% and 80%, and 65% and 70%, respectively [25]. The increased MPI is also associated with intrauterine hypoxia which leads to redistribution of blood circulation in FGR [26], and cerebral vasodilation further lead to abnormal left and right ventricular cardiac blood flow output, which exacerbates cardiac abnormalities in FGR [27]. Ductus venosus is not only the main distributor of fetal oxygenated blood flow, but also the direct channel between peripheral vein and central venous system. Its change can indirectly evaluate the degree of fetal intrauterine hypoxia [28]. In our study, we found that ductus venosus S/a increased significantly in FGR group, which may be related to the decline of cardiac diastolic function, the increase of venous ductus reflux resistance and the decrease of blood flow in FGR. In addition, S/a in predicting the incidence of FGR yielded AUC of 0.784. The study presented by Yin et al. [29] showed that lower value of S/D, PI, and RI of UA, and higher value of S/D, PI, and RI of MCA were associated with good pregnancy outcomes. The univariate analysis of the present study also indicated the poor pregnancy outcomes were related to higher value of MPI, S/D, RI, PI of UA, and S/a, as well as the lower scores of 1 min Apgar, along with lower values regarding S/D, RI, and PI of MCA. Furthermore, these values were applied to predict the incidence of poor pregnancy outcomes in FGR, and the MPI, S/D, RI, PI of UA, S/D, RI, PI of MCA, and S/a yielded AUC of 0.806, 0.833, 0.774, 0.788, 0.807, 0.729, 0.748, and 0.770. It shows that determination of UA, MCA, and ductus venosus Doppler blood flow spectrum can provide scientific guidance for clinical prediction of pregnancy outcome of FGR. The Apgar score is a convenient and rapid method for revealing the status of the newborn infant immediately following birth. It has been reported that low 5 minutes Apgar score is associated with short-term infant morbidity and mortality [30], as well as an increased risk of long-term pediatric gastro-intestinal morbidity of the offspring [31] In our study, the Pearson correlation coefficients manifested that S/D, RI, and PI of MCA were positively correlated with 1 min Apgar scores, while MPI, S/D, RI, PI of UA, and S/a were negatively correlated with the 1 min Apgar score. These outcomes emphasize the importance of MPI, blood flow spectrum of UA, MCA, and ductus venosus on pregnancy outcomes.

The article "Prenatal Prediction of Fetal Growth Restriction and Postnatal Outcomes by Ultrasound Assessment of Fetal Myocardial Performance Index and Blood Flow Spectrum" was retracted in 2023. Reasons: suspected computer-generated content; unreliable results or conclusions; concerns about the data; concerns about the results or conclusions.

In conclusion, the MPI value, the parameters of blood flow spectrum of UA, MCA, and ductus venosus increased, while MCA blood flow spectrum parameters decreased in FGR. These changes are helpful to guide the clinical prediction of FGR and its pregnancy outcomes. Considering the modest sample size, only FGR pregnant women and healthy pregnant women included, potentially, and retrospective nature of this study, further investigations in a cohort of singleton SGA/FGR fetuses seem to be required.

## Figures and Tables

**Figure 1:** ROCs of MPI, S/D, RI, PI of UA and MCA, and S/a used to predict the incidence of FGR.

**Figure 2:** ROCs of MPI, S/D, RI, PI of UA and MCA, and S/a used to predict the incidence of poor pregnancy outcomes for pregnant women developing FGR.

**Table 1:** MPI, S/D, RI, PI of UA and MCA, and S/a between the FGR group and the control group.

Parameter	Control group (*n* = 242)	FGR group (*n* = 242)	*P*
MPI	0.43 ± 0.05	0.50 ± 0.06	<0.001

UA blood flow			
S/D	2.63 ± 0.53	3.42 ± 0.57	<0.001
RI	0.60 ± 0.18	0.79 ± 0.15	<0.001
PI	0.83 ± 0.27	1.14 ± 0.22	<0.001

MCA blood flow			
S/D	3.96 ± 0.88	2.81 ± 0.87	<0.001
RI	0.82 ± 0.20	0.58 ± 0.18	<0.001
PI	1.59 ± 0.34	1.21 ± 0.28	<0.001
S/a	1.99 ± 0.43	2.51 ± 0.45	<0.001

Results were compared by independent sample *t*-test.

The article "Prenatal Prediction of Fetal Growth Restriction and Postnatal Outcomes by Ultrasound Assessment of Fetal Myocardial Performance Index and Blood Flow Spectrum" was retracted in 2023. Reasons: suspected computer-generated content; unreliable results or conclusions; concerns about the data; concerns about the results or conclusions.

**Table 2:** AUCs with 95%CI and cutoff values of MPI, S/D, RI, PI of UA and MCA, and S/a used to predict the incidence of FGR.

Parameter	AUC	95%CI	*P*	Cutoff values
MPI	0.813	0.776–0.850	<0.001	0.47

UA blood flow				
S/D	0.835	0.798–0.873	<0.001	2.93
RI	0.791	0.748–0.833	<0.001	0.70
PI	0.804	0.765–0.843	<0.001	1.02

MCA blood flow				
S/D	0.789	0.747–0.830	<0.001	3.28
RI	0.796	0.755–0.837	<0.001	0.68
PI	0.803	0.761–0.845	<0.001	1.35
S/a	0.784	0.742–0.826	<0.001	2.22

**Table 3:** MPI, S/D, RI, PI of UA and MCA, and S/a between pregnant women with poor pregnancy outcomes and those with favorable pregnancy outcomes.

Parameter	Poor pregnancy outcomes (*n* = 33)	Favorable pregnancy outcomes (*n* = 209)	*P*
MPI	0.56 ± 0.05	0.49 ± 0.05	<0.001

UA blood flow			
S/D	3.96 ± 0.38	3.34 ± 0.55	<0.001
RI	0.92 ± 0.11	0.77 ± 0.15	<0.001
PI	1.33 ± 0.18	1.11 ± 0.21	<0.001

MCA blood flow			
S/D	2.23 ± 0.17	2.90 ± 0.90	<0.001
RI	0.47 ± 0.07	0.60 ± 0.19	<0.001
PI	1.02 ± 0.14	1.24 ± 0.28	<0.001
S/a	2.86 ± 0.22	2.46 ± 0.45	<0.001
1 min Apgar score	6.25 ± 0.44	8.90 ± 0.55	<0.001

Results were compared by independent sample *t*-test.

**Table 4:** AUCs with 95%CI and cutoff values of MPI, S/D, RI, PI of UA and MCA, and S/a used to predict the incidence of poor pregnancy outcomes for pregnant women developing FGR.

Parameter	AUC	95%CI	*P*	Cutoff values
MPI	0.806	0.727–0.885	<0.001	0.50

UA blood flow				
S/D	0.833	0.767–0.900	<0.001	3.51
RI	0.774	0.690–0.859	<0.001	0.82
PI	0.788	0.710–0.866	<0.001	1.14

MCA blood flow				
S/D	0.807	0.735–0.880	<0.001	2.44
RI	0.729	0.654–0.803	<0.001	0.53
PI	0.748	0.671–0.826	<0.001	1.14
S/a	0.770	0.698–0.841	<0.001	2.64

## Data Availability

The data used to support the findings of this study are included within the article.
